# Laparoscopic vs. Open Pancreaticoduodenectomy After Learning Curve: A Systematic Review and Meta-Analysis of Single-Center Studies

This article has been retracted.

**DOI:** 10.3389/fsurg.2021.715083

**Published:** 2021-09-10

**Authors:** Qingbo Feng, Zechang Xin, Jie Qiu, Mei Xu

**Affiliations:** ^1^Department of Liver Surgery and Liver Transplantation Centre, West China Hospital, Sichuan University, Chengdu, China; ^2^Key Laboratory of Carcinogenesis and Translational Research (Ministry of Education/Beijing), Department of Hepatobiliary and Pancreatic Surgery Unit I, Peking University Cancer Hospital & Institute, Beijing, China; ^3^Affiliated Hospital of Zunyi Medical University, Zunyi, China; ^4^Department of Ultrasound Diagnosis, Air Force Medical Centre, Beijing, China

**Keywords:** pancreatic cancer, pancreaticoduodenectomy, laparoscopic, whipple, meta-analysis

## Abstract

**Background:** Although laparoscopic pancreaticoduodenectomy (LPD) is a safe and feasible treatment compared with open pancreaticoduodenectomy (OPD), surgeons need a relatively long training time to become technically proficient in this complex procedure. In addition, the incidence of complications and mortality of LPD will be significantly higher than that of OPD in the initial stage. This meta-analysis aimed to compare the safety and overall effect of LPD to OPD after learning curve based on eligible large-scale retrospective cohorts and randomized controlled trials (RCTs), especially the difference in the perioperative and short-term oncological outcomes.

**Methods:** PubMed, Web of Science, EMBASE, Cochrane Central Register, and ClinicalTrials.gov databases were searched based on a defined search strategy to identify eligible studies before March 2021. Only clinical studies reporting more than 40 cases for LPD were included. Data on operative times, blood loss, and 90-day mortality, reoperation, length of hospital stay (LOS), overall morbidity, Clavien–Dindo ≥III complications, postoperative pancreatic fistula (POPF), blood transfusion, delayed gastric emptying (DGE), postpancreatectomy hemorrhage (PPH), and oncologic outcomes (R0 resection, lymph node dissection, positive lymph node numbers, and tumor size) were subjected to meta-analysis.

**Results:** Overall, the final analysis included 13 retrospective cohorts and one RCT comprising 2,702 patients (LPD: 1,040, OPD: 1,662). It seems that LPD has longer operative time (weighted mean difference (WMD): 74.07; 95% CI: 39.87–108.26; *p* < 0.0001). However, compared with OPD, LPD was associated with a higher R0 resection rate (odds ratio (OR): 1.43; 95% CI: 1.10–1.85; *p* = 0.008), lower rate of wound infection (OR: 0.35; 95% CI: 0.22–0.56; *p* < 0.0001), less blood loss (WMD: −197.54 ml; 95% CI −251.39 to −143.70; *p* < 0.00001), lower blood transfusion rate (OR: 0.58; 95% CI 0.43–0.78; *p* = 0.0004), and shorter LOS (WMD: −2.30 day; 95% CI −3.27 to −1.32; *p* < 0.00001). No significant differences were found in 90-day mortality, overall morbidity, Clavien–Dindo ≥ III complications, reoperation, POPF, DGE, PPH, lymph node dissection, positive lymph node numbers, and tumor size between LPD and OPD.

**Conclusion:** Comparative studies indicate that after the learning curve, LPD is a safe and feasible alternative to OPD. In addition, LPD provides less blood loss, blood transfusion, wound infection, and shorter hospital stays when compared with OPD.

## Introduction

Pancreaticoduodenectomy (PD) is a very complex procedure that can provide a cure or prolonged survival for benign lesions and cancer in the periampullary region and pancreatic head (1). Laparoscopic pancreaticoduodenectomy (LPD) and open pancreaticoduodenectomy (OPD) are the two treatment modalities for pancreatic and periampullary malignancies and some benign diseases, with the former offering the better results in terms of blood loss and hospital stay. OPD is a conventional procedure. But since Gagner and Pomp reported LPD in 1994, (2) LPD is increasingly used worldwide, but only 285 reported cases have been reported as of 2011 and the safety and feasibility of LPD remain controversial (3).

Over the last decade, laparoscopic surgery has emerged as a viable alternative approach to conventional open surgery and emphasized that it is superior to OPD in reducing blood loss, shorter hospital stay, earlier oral intake, less pain, and faster recovery (4–7). However, an analysis of 983 patients found that patients who underwent LPD had higher 30-day mortality compared to those with OPD in low-volume centers (8). Although LPD has the potential advantages of a lower degree of invasion, fast recovery, less pain, and excellent vision, surgeons need a relatively long training time to become technically proficient in this complex procedure. Therefore, given this condition, there is still no consensus among pancreatic surgeons on whether the gold standard for pancreatic head cancer or (and) periampullary malignancies is LPD or open approach.

As with all surgical studies, the experience and performance of surgeons have a significant impact on outcomes which can be a source of bias. Furthermore, the great majority of the studies on LPD and OPD are small sample study and the surgeons remained in the early training phase. Wang et al. and Zhang et al. showed that a minimum of 40 cases are required for surgeons to make LPD become stable (9, 10). In addition, even at experienced, high-volume centers, the surgical results during the learning curve are not satisfactory (11, 12). Therefore, to find a better approach for patients with pancreatic head cancer or (and) periampullary malignancies and some benign diseases, we used data from good quality articles to conduct a systematic review and meta-analysis to compare the clinical outcomes of LPD vs. OPD after the learning curve.

## Methods

### Materials and Methods

This study has been reported in line with the recommendations of the PRISMA guidelines (13) and registered at PROSPERO with registration number: CRD42021246730. This article is a meta-analysis; therefore, Institutional Review Board approval is not needed for this study.

### Data Sources and Search Strategy

Published studies were systematically searched in PubMed, Web of Science, EMBASE, Cochrane Central Register, and ClinicalTrials.gov databases before March 15, 2021, by two independent investigators (QB Feng, ZC Xin). The following key terms and their combinations were used: laparoscopic, open, conventional, Whipple, and pancreaticoduodenectomy. To prevent missing relevant publications, computer search was supplemented with manual searches of the references of publications and reviews.

### Inclusion and Exclusion Criteria

Two investigators (QB Feng, ZC Xin) reviewed the currently available literature and screened all abstracts and titles independently and determined eligible studies based on the following criteria.

Inclusion criteria were as follows: (1) types of interventions: LPD and OPD; (2) types of studies: randomized controlled trials (RCTs), retrospective studies, cohort studies, and case-control studies; (3) sample size: LPD > 40; (4) study from a single-center; and (5) primary article published in English.

Exclusion criteria were as follows: (1) non-English studies; (2) insufficient information available in the abstracts; (3) data that were incomplete; and (4) editorials, letters, non-human studies, expert opinions, reviews, case reports, and studies without control groups.

### Data Extraction and Quality Assessment

Two reviewers (QB Feng, ZC Xin) extracted the original data independently using a unified datasheet, and in the case of any ambiguity, a third observer (J Qiu) was consulted to review the study to reach a consensus. Data extraction included the following items: study and patient characteristics, operative and postoperative outcomes. Study and patient characteristics included first author, country, publication year, research design, sample size, and mean age; the latter included operative time, blood loss, blood transfusion, tumor size, postoperative morbidity and 90-day mortality, length of hospital stay (LOS), R0 resections, and several harvested lymph nodes. The Newcastle–Ottawa scale was used to assess the quality of included studies by two different assessors.

Each study was scored between 0 and 9 according to Newcastle-Ottawa Scale (NOS), a score of ≥6 is considered indicative of high quality. Two reviewers (QB Feng, ZC Xin) assessed the included studies independently (14).

### Statistical Analysis

Review Manager 5.3 software was used to analyze data. Odds ratio (OR) and weighted mean difference (WMD) with the 95% CI were used for the assessment of dichotomous and continuous variables, respectively. We adopted the method described by Hozo et al. to calculate the mean values and SD (15). A funnel plot was used to assess potential publication bias. Statistical heterogeneity was quantified using Higgin's I^2^ index. A study with an I^2^ < 50% was considered indicative of low or moderate heterogeneity, and the fixed effect mode (FEM) was then applied to pool the results. A study with an I^2^ > 50% was considered a high heterogeneity and the random effect model (REM) was adopted.

## Results

### Search Results and Characteristics of the Included Studies

The literature search yielded 556 relevant English publications from various electronic databases. According to the inclusion criteria, 13 retrospective cohort studies and one RCT (5, 7, 16–27) comparing LPD and OPD in a total of 2,702 patients (1,040 and 1,662 underwent LPD and OPD, respectively) were included for further analysis. A flow chart of our analysis protocol is shown in Figure 1. The major features and qualities of these 14 studies are listed in Table 1, while the assessment of the risk of bias in individual studies made with the Cochrane risk of bias tool is presented as a summary in Figure 2. All results of this meta-analysis are presented in Table 2.

**Figure 1:** Flow chart of study identification and selection.

**Table 1:** Characteristics of included studies.

**Author-Year**	**Country**	**Study Type**	**Study Interval**	**Samples**		**Age (mean ± SD)**		**Sex (M/F)**		**BMI (mean ± SD)**	
				**LPD**	**OPD**	**LPD**	**OPD**	**LPD**	**OPD**	**LPD**	**OPD**
Asbun et al. 2012 (16)	USA	RS	2005–2011	53	215	62.9 ± 14.14	67.3 ± 11.53	29/24	95/120	27.64 ± 7.16	26.6 ± 5.08
Mesleh et al. 2013 (17)	USA	RS	2009–2012	75	48	NA	NA	43/32	23/25	NA	NA
Croome et al. 2014 (7)	USA	RS	2008–2013	108	214	66.6 ± 9.6	65.4 ± 10.9	51/57	131/83	27.4 ± 5.4	27.2 ± 5.3
Dokmak et al. 2015 (18)	France	RS	2011–2014	46	46	60 (27–85)	63 (47–81)	26/20	28/18	22.6 (17–30)	26.4 (19–42)
Song et al. 2015 (5)	South Korea	RS-PSM	2007–2012	93	93	49.6 ± 13.4	50.1 ± 13	47/46	47/46	22.8 ± 2.7	23.1 ± 2.5
Stauffer et al. 2016 (19)	USA	RS	1995–2014	58	193	69.9 (40.6–84.8)	68.9 (33.3–86.9)	32/26	96/97	25.9 (17.7–49.6)	25.6 (15.0–46.1)
Delitto et al. 2016 (20)	USA	RS	2010–2014	52	50	65.3 ± 1.7	68.6 ± 1.4	34/18	28/22	26.3 ± 0.8	25.5 ± 0.7
Kuesters et al. 2018 (21)	Germany	RS	2010–2016	62	278	71	68	31/31	137/141	24.7 (15–39)	24.7 (16–46)
Han et al. 2019 (22)	Korea	RS-PSM	2012–2017	87	87	65.1± 8.8	63.6± 9.5	49/38	53/34	23.52 ± 2.74	23.32 ± 3.08
Hilst et al. 2019 (23)	Netherland	RCT	2016–2017	50	49	67 (59–76)	66 (61–73)	20/30	25/24	25 ± 3	26 ± 4
Kim et al. 2019 (24)	Korea	RS	2016–2017	58	91	49.5 ± 12.0	56.0 ± 10.5	18/40	42/49	23.1 ± 2.5	24.5 ± 3.6
Yoo et al. 2020 (25)	Korea	RS-PSM	2011–2017	69	69	62.8 ± 10.1	63.2 ± 8.6	34/35	38/31	23.1 ± 2.7	23.5 ± 3.3
Dang et al. 2020 (26)	China	RS-PSM	2011–2019	131	131	57.41 ± 9.42	57.52 ± 9.50	81/50	79/52	21.71 ± 2.81	21.67 ± 2.98
Huang et al. 2020 (27)	China	RS-PSM	2016–2019	98	98	57.47 ± 13.0	59.09 ± 11.5	54/44	56/42	24.5 ± 3.12	25.1 ± 2.26

*LPD, laparoscopic pancreaticoduodenectomy; OPD, open pancreaticoduodenectomy; M/F, male/female; SD, standard deviation; BMI, body mass index; NA, not applicable*.

**Figure 2:** Quality assessment of included studies. Overall (left) and study-level risk of bias (right), using Cochrane risk of the bias assessment tool. Studies were deemed to be at high, low, or unclear risk of bias based on the adequacy of sequence generation, allocation concealment, blinding, method of addressing incomplete data, selective reporting, and other biases. The review judgments of authors about each risk of bias item are presented as percentages across all included studies and for each included study.

**Table 2:** Summary results of the meta-analyses.

**Outcomes of interest**	**Studies, n**	**LPD**	**OPD**	**WMD/OR(95%CI)**	***P*** **value**	**Heterogeneity**			
						**X^2^**	**df**	**I^2^,%**	***P*** **value**
Length of stay (day)	14	1,040	1,662	74.07(39.87,108.26)	*P* < 0.0001	1,769.74	12	99	*P* < 0.00001
Blood loss (ml)	11	834	1,267	−197.54(−251.39,−143.70)	*P* < 0.00001	251.34	10	96	*P* < 0.00001
Blood transfusion	7	493	948	0.58(0.43,0.78)	*P* = 0.0004	4.90	6	0	*P* = 0.56
Operative time (min)	14	1,040	1,662	−2.3(−3.27,−1.32)	*P* < 0.00001	67.73	13	81	*P* < 0.00001
Overall complication rates	10	753	1,135	0.89(0.73,1.09)	*P* = 0.25	14.28	9	37	*P* = 0.11
Clavien-Dindo grade ≥ III	8	546	789	1(0.62,1.64)	*P* = 0.99	17.92	7	61	*P* = 0.01
90-days mortality	5	431	809	0.91(0.51,1.62)	*P* = 0.74	4.82	4	17	*P* = 0.31
Postpancreatectomy hemorrhage	7	539	939	1.14(0.74,1.77)	*P* = 0.54	2.77	6	0	*P* = 0.84
Wound infection	5	311	605	0.35(0.22,0.56)	*P* < 0.0001	3.24	4	0	*P* = 0.52
Postoperative pancreatic fistula	13	979	1,384	0.83(0.67,1.03)	*P* = 0.09	18.77	12	36	*P* = 0.09
Delayed gastric emptying	12	927	1,334	−0.03(−0.06,0.00)	*P* = 0.08	16.28	11	32	*P* = 0.13
Reoperation	10	719	1,236	0.97(0.62,1.5)	*P* = 0.88	9.99	9	10	*P* = 0.35
R0 resection rate	11	827	1,475	1.43(1.1,1.85)	*P* = 0.008	12.84	10	22	*P* = 0.23
Lymph nodes harvested	10	739	1,388	0.87(−0.27,2.02)	*P* = 0.13	118.87	9	92	*P* < 0.00001
Positive lymph node numbers	3	163	356	−0.07(−0.16,0.02)	*P* = 0.14	0.89	2	0	*P* = 0.64
Tumor size	11	741	1,390	−0.13(−0.42,0.15)	*P* = 0.35	126.42	10	92	*P* < 0.00001

*LPD, laparoscopic pancreaticoduodenectomy; OPD, open pancreaticoduodenectomy; WMD, weighted mean difference; OR, odds ratio; CI, confidence interval*.

### Operative Outcomes

#### Operative Time

Fourteen studies (5, 7, 16–27) with a total of 2,702 patients (1,040 patients who underwent LPD and 1,662 patients who underwent OPD) reported operative times. We found that operative time was longer in the LPD group (WMD: 74.07 min; 95% CI: 39.87–108.26; *p* < 0.00001). Heterogeneity was high (I^2^ = 99%) and analyzed in the REM (Figure 3A).

**Figure 3:** Forest plot of comparison of LPD vs. OPD for operative outcomes. **(A)** Forest plot for the length of stay; **(B)** forest plot for blood loss; and **(C)** forest plot for blood transfusion.

#### Blood Loss

Estimated blood loss was assessed in 11 studies (5, 7, 16, 18–20, 22–24, 26, 27). The pooled data revealed that blood loss was lesser in LPD group (WMD: −197.54 ml; 95% CI: −251.39 to −143.70; *p* < 0.00001). Heterogeneity was high (I^2^ = 96%) and analyzed in REM (Figure 3B).

#### Blood Transfusion

Blood transfusion rate data were available in seven studies (7, 18–21, 25, 26). The meta-analysis suggested blood transfusion rate was higher in the OPD group (OR: 0.58; 95% CI: 0.43–0.78; *p* = 0.0004). Heterogeneity was not significant (I^2^ = 0%) and analyzed in FEM (Figure 3C).

### Postoperative Outcomes

#### Length of Stay

All studies (5, 7, 16–27) with a total of 2,702 patients (1,040 patients who underwent LPD and 1,662 patients who underwent OPD) investigated the LOS. The meta-analysis suggested a shorter LOS in the LPD group (MD = −2.30; 95% CI: −3.27 to −1.32; *p* < 0.00001) (Figure 4A).

**Figure 4:** Forest plot of comparison of LPD vs. OPD for postoperative outcomes. **(A)** Forest plot for operative time; **(B)** forest plot for overall complication rates; **(C)** forest plot for Clavien–Dindo grade ≥ III; and **(D)** forest plot for 90-day mortality.

#### Overall Complication Rates

Ten studies (5, 18, 19, 21–27) that encompassed 1,888 patients (753 patients and 1,135 patients underwent LPD and OPD, respectively), recorded the postoperative complications, and the present analysis revealed no significant differences between the two groups (OR: 0.89; 95% CI: 0.73–1.06; *p* = 1.09). The heterogeneity was low (I^2^ = 37%) and analyzed in FEM (Figure 4B).

#### Clavien–Dindo Grade ≥ III

Eight studies (7, 17–20, 23, 24, 26) with a total of 1,335 patients (546 patients and 789 patients underwent LPD and OPD, respectively) reported the Clavien–Dindo classifications of complications according to Dindo et al. (28) No significant differences in Clavien–Dindo grade ≥III were observed between these two groups (OR: 1.00; 95% CI: 0.62–1.64; *p* = 0.99). The heterogeneity was high (I^2^ = 61%) and analyzed in the REM (Figure 4C).

#### 90-Day Mortality

Pooling the data from five studies (16, 21, 22, 26, 27) that included 1,240 patients (431 patients and 809 patients underwent LPD and OPD, respectively) assessed the 90-day mortality. The pooled data showed no differences in 90-day mortality (OR: 0.91; 95% CI: 0.51–1.62; *p* = 0.74), with low heterogeneity (I^2^ = 17%) in FEM (Figure 4D).

#### Postpancreatectomy Hemorrhage

Pooling the data of seven studies (7, 16, 19, 20, 22, 23, 27) that included 1,478 patients (539 patients who underwent LPD and 939 patients who underwent OPD) assessed postpancreatectomy hemorrhage, and the present analysis revealed no significant differences in postpancreatectomy hemorrhage (WMD: 1.14; 95% CI: 0.74–1.77; *p* = 0.54), with a low heterogeneity (I^2^ = 0%) in the FEM (Figure 5A).

**Figure 5:** Forest plot of comparison of LPD vs. OPD for overall complication rates. **(A)** Forest plot for postpancreatectomy hemorrhage; **(B)** forest plot for wound infection; **(C)** forest plot for postoperative pancreatic fistula; **(D)** forest plot for delayed gastric emptying; and **(E)** forest plot for reoperation.

#### Wound Infection

Five studies (16, 19, 20, 23, 26) with a total of 916 patients (311 patients who underwent LPD and 605 patients who underwent OPD) reported the wound infection rate, and the pooled data revealed a significant lower wound infection rate in the LPD group (OR: 0.35; 95% CI: 0.22–0.56; *p* < 0.0001), with no heterogeneity (I^2^ = 0%) in FEM (Figure 5B).

#### Postoperative Pancreatic Fistula

Postoperative pancreatic fistula (POPF) incidence rates were described for 2,363 patients in 13 studies (5, 7, 16–20, 22–27). No significant differences in POPF rates were observed between these two groups (OR: 0.83; 95% CI: 0.67–1.03; *p* = 0.09), with a low heterogeneity (I^2^ = 36%) in FEM (Figure 5C).

#### Delayed Gastric Emptying

Twelve studies (5, 7, 16–19, 22–27) with a total of 2,261 patients (927 patients who underwent LPD and 1,334 patients who underwent OPD) reported delayed gastric emptying (DGE) rate, and the result of meta-analysis indicated no difference in DGE (OR: −0.03; 95% CI: −0.06 to 0.00; *p* = 0.08), with a moderate heterogeneity (I^2^ = 32%) in FEM (Figure 5D).

#### Reoperation

Ten studies (16–19, 21–24, 26, 27) with a total of 1,955 patients (719 patients who underwent LPD and 1,236 patients who underwent OPD) reported the incidence of reoperation, and the pooled data revealed no difference in reoperation (OR: 0.97; 95% CI: 0.62–1.50; *p* = 0.88), with low heterogeneity (I^2^ = 10%) in FEM (Figure 5E).

### Short-Term Oncological Outcomes

#### R0 Resection Rate

In total, 11 studies including 2,302 patients (827 patients who underwent LPD and 1,475 patients who underwent OPD) provided data regarding the R0 resection rate (16–24, 26, 27). We found that LPD was associated with a higher R0 resection rate (OR: 1.43; 95% CI: 1.10–1.85; *p* = 0.008), with low heterogeneity (I^2^ = 22%) as shown in the FEM (Figure 6A).

**Figure 6:** Forest plot of comparison of LPD vs. OPD for short-term oncological outcomes. **(A)** Forest plot for R0 resection rate; **(B)** forest plot for lymph node dissection; **(C)** forest plot for positive lymph node number; and **(D)** forest plot for tumor size.

#### Lymph Node Dissection

Ten studies (7, 16, 19–21, 23–27) including 2,127 patients (739 patients who underwent LPD and 1,388 patients who underwent OPD) assessed the number of lymph node dissection, the result of meta-analysis revealed no difference in lymph node dissection (WMD: 0.87; 95% CI: −0.27 to 2.02; *p* = 0.13), with a high heterogeneity (I^2^ = 92%) in the REM (Figure 6B).

#### Positive Lymph Node Numbers

Three studies (16, 20, 24) that included 519 patients (163 patients who underwent LPD and 356 patients who underwent OPD) assessed positive lymph node numbers, the result of meta-analysis revealed no difference in positive lymph node numbers (WMD: −0.07; 95% CI: −0.16 to 0.02; *p* = 0.14), with no heterogeneity (I^2^ = 0%) in the FEM (Figure 6C).

#### Tumor Size

Eleven studies (7, 16, 18–26) that included 2,131 patients (741 patients who underwent LPD and 1,390 patients who underwent OPD) assessed the tumor size, the result of meta-analysis showed no statistically significant difference between the LPD and OPD groups (WMD: −0.13; 95% CI: −0.42 to 0.15; *p* = 0.35), with no heterogeneity (I^2^ = 92%) in the REM (Figure 6D).

#### Publication Bias

Begg's funnel plot was drawn for each outcome and used to assess publication bias. As shown in the funnel plot of the R0 rate (Figure 7), all studies that lie inside the 95% CIs indicated no publication bias.

**Figure 7:** Funnel plots for postoperative pancreatic fistula.

## Discussion

Laparoscopic pancreatoduodenectomy (LPD) is considered as the “Everest” of abdominal endoscopic surgery due to its complicated operation process and high requirements for surgeons. The special anatomy structure, complicated vascular variation, various and critical postoperative complications, and extremely difficult operation in the pancreas restrict the further development of LPD. Since 2011, with the accumulation of laparoscopic experience, and the replacement of laparoscopic equipment and instruments, LPD has been developed rapidly and widely carried out in large medical centers at home and abroad. Pancreatectomy and alimentary tract reconstruction in laparoscopic are the key points for LPD. Therefore, the surgeons should have sufficient open surgery experience and excellent laparoscopic skills. At present, only a few large hepatobiliary and pancreatic centers routinely carry out LPD at home and abroad. Since LPD is one of the most complex laparoscopic operations in the field of general surgery, it has the characteristics of a long learning curve and high risk. If the quality cannot be effectively controlled during the initial stage, the incidence of complications and mortality of LPD will be significantly higher than that of open surgery. Wang et al. and Zhang et al. showed that pancreatic surgeons need a minimum of 40 cases to be proficient at LPD (9). According to Wang et al.'s study, the LPD learning curve can be divided into an initial stage, technical competence stage, and challenging period stage (9). In addition, after the learning curve of LPD, the prognosis of patients can be improved with the improvement of proficiency. To compare the real difference between LPD and OPD, we analyzed the data from the literature that LPD included more than 40 cases from a single-center. Finally, 13 large-scale retrospective cohorts and one RCT consisting of 2,702 patients were included in this study to compare the perioperative outcomes and oncologic outcomes and of LPD with OPD after the learning curve.

To the best of our knowledge, this is the first meta-analysis to evaluate the safety and overall effect of LPD on OPD after the learning curve. The results of our meta-analysis show that LPD has a shorter LOS, lower wound infection rate, less blood loss but a longer operative time than OPD, which was similar to the study of Yin et al. (29) LPD has a longer operative time as a result of longer pancreatectomy and digestive tract reconstruction under laparoscope.

Negative margin and the number of lymph node dissection are two important malignancy prognosis factors in PD. Pooled data from this meta-analysis revealed that LPD has a higher R0 rate than OPD. We think that this may be explained by patients with early-stage or even benign diseases who were selected to perform LPD. From the perspective of tumor radical effect, the results of this study show that the two surgical methods have the same effect in the number of lymph node dissections, suggesting that LPD and OPD have the same tumor radical effect, which is consistent with the results of the most existing clinical studies (5, 30).

With the improvement of pancreatic surgery technology, postoperative mortality has decreased, but postoperative complications are still high, which is still a difficult problem for surgeons. There are many complications of LPD, namely, pancreatic fistula, postoperative bleeding, gastric emptying disorder, wound infection, wound dehiscence, pneumonia, respiratory failure, urinary tract infection, stroke, renal failure, cardiac arrest, myocardial infarction, thromboembolic events, septic shock, sepsis, reoperation, etc. Among them, pancreatic fistula is one of the most important complications after pancreatic surgery. Pancreatic fistula can lead to a prolonged hospital stay, increased treatment costs, and even life-threatening. With the improvement of surgeon technology, the incidence of complications is decreasing. The study used the pancreatic fistula rate to evaluate the effect of a learning curve on LPD complications and confirmed the relationship between proficiency and complications.

The present study shows that there was no significant difference in the 90-day mortality, overall complication rates, POPF, and the incidence of severe complications (Clavien–Dindo III/IV grade complications) between the two groups, indicating that after the learning curve LPD is as safe as OPD. POPF was considered the most common and difficult complication as a result of causing DGE, hemorrhage, and influence postoperative mortality. (31, 32) At present, most studies have confirmed that the incidence of pancreatic fistula in LPD and OPD is similar, and the difference is not statistically significant. Postoperative bleeding may come from the anastomotic stoma, blood vessels, pancreatic stump, stress ulcer, etc.

To evaluate the safety and efficiency of LPD, this meta-analysis included 14 studies and showed that LPD was comparable with OPD. However, there are still some limitations in this study. First, the main limitation is that most of the included studies were retrospective research and there was only one RCT, which may have contributed to selection bias. Second, none of the studies has evaluated the long-term outcomes, which limits our ability to draw useful prognostic conclusions and quality of life. Furthermore, some eligible studies included benign diseases that may affect the prognosis of patients. Therefore, further large-scale prospective comparative studies and RCTs are expected to provide more convincing results for evaluation to further analyze the safety and efficacy of LPD after the learning curve is expected to solve these limitations.

## Conclusion

This systematic review and meta-analysis suggested that after the learning curve LPD is a safe alternative to OPD, as it is associated with significant reductions in blood loss, blood transfusion, LOS, wound infection rate, and higher R0 rate. Furthermore, high-quality RCTs with survival outcomes are expected to further assess the safety and efficiency of LPD after the learning curve.

## Data Availability Statement

The raw data supporting the conclusions of this article will be made available by the authors, without undue reservation.

## Author Contributions

QF study concept and design. QF and ZX acquisition of data. QF, ZX, and JQ analysis and interpretation of data. QF and ZX drafting of the manuscript. MX critical revision of the manuscript for important intellectual content, administrative, technical, or material support, and study supervision. All authors contributed to the article and approved the submitted version.

## Conflict of Interest

The authors declare that the research was conducted in the absence of any commercial or financial relationships that could be construed as a potential conflict of interest.

## Publisher's Note

All claims expressed in this article are solely those of the authors and do not necessarily represent those of their affiliated organizations, or those of the publisher, the editors and the reviewers. Any product that may be evaluated in this article, or claim that may be made by its manufacturer, is not guaranteed or endorsed by the publisher.
